RETRACTED

# Extreme Resistance as a Host Counter-counter Defense against Viral Suppression of RNA Silencing

**DOI:** 10.1371/journal.ppat.1003435

**Published:** 2013-06-13

**Authors:** Raphaël Sansregret, Vanessa Dufour, Mathieu Langlois, Fouad Daayf, Patrice Dunoyer, Olivier Voinnet, Kamal Bouarab

**Affiliations:** 1 Centre SEVE, Département de Biologie, Faculté des Sciences, Université de Sherbrooke, Sherbrooke, Quebec, Canada; 2 Department of Plant Science, University of Manitoba, Winnipeg, Manitoba, Canada; 3 Institut de Biologie Moléculaire des Plantes du CNRS, Université de Strasbourg, Strasbourg, France; 4 Department of Biology, Swiss Federal Institute of Technology (ETH), Zurich, Switzerland; University of California Riverside, United States of America

## Abstract

RNA silencing mediated by small RNAs (sRNAs) is a conserved regulatory process with key antiviral and antimicrobial roles in eukaryotes. A widespread counter-defensive strategy of viruses against RNA silencing is to deploy viral suppressors of RNA silencing (VSRs), epitomized by the P19 protein of tombusviruses, which sequesters sRNAs and compromises their downstream action. Here, we provide evidence that specific *Nicotiana* species are able to sense and, in turn, antagonize the effects of P19 by activating a highly potent immune response that protects tissues against *Tomato bushy stunt virus* infection. This immunity is salicylate- and ethylene-dependent, and occurs without microscopic cell death, providing an example of “extreme resistance” (ER). We show that the capacity of P19 to bind sRNA, which is mandatory for its VSR function, is also necessary to induce ER, and that effects downstream of P19-sRNA complex formation are the likely determinants of the induced resistance. Accordingly, VSRs unrelated to P19 that also bind sRNA compromise the onset of P19-elicited defense, but do not alter a resistance phenotype conferred by a viral protein without VSR activity. These results show that plants have evolved specific responses against the damages incurred by VSRs to the cellular silencing machinery, a likely necessary step in the never-ending molecular arms race opposing pathogens to their hosts.

## Author Summary

Multiple and complex layers of defense help plants to combat pathogens. A first line of defense relies on the detection, via dedicated host-encoded receptors, of signature molecules (so called pathogen-associated molecular patterns, PAMPs) produced by pathogens. In turn, this PAMP-triggered immunity (PTI) may be itself antagonized by adapted pathogens that have evolved virulence effectors to target key PTI components. Host plants react to PTI suppression by producing disease resistance (R) proteins that recognize virulence effectors and activate highly specific resistance called Effector Triggered Immunity (ETI). It has been noted that RNA silencing, a sequence-specific antiviral defense response based on the production of virus-derived 21–24 nt small RNAs on the one hand, and its suppression by virulence effectors, called viral suppressors of RNA silencing (VSRs) on the other, are conceptually similar to PTI. Here we provide strong support to this hypothesis by showing that extreme resistance is indeed activated following detection, in specific host species, of the VSR activity of a viral virulence effector. The ensuing antiviral immunity displays many characteristics of ETI, suggesting that one or several R proteins must sense the integrity of the host silencing machinery.

RETRACTED

## Introduction

Plants fight microbial attacks using both constitutive and induced defenses, which include basal and highly specific resistance [1]. Basal resistance, or PTI (for PAMP-Triggered Immunity), often relies on the detection of highly conserved signature molecules that include fungal polysaccharides or bacterial flagellin, collectively termed pathogen-associated molecular patterns (PAMPs; [1], [2]). To circumvent this first layer of defense, many host-adapted microbes produce effector proteins that suppress various steps of PTI [3]. As a counter-response, plants have, in turn, evolved classes of specialized receptors called resistance (R) proteins that directly detect pathogen's encoded suppressors of PTI, or that sense the molecular consequences of their adverse action on defense-related host factors.

R protein activation triggers potent defense responses collectively named Effector Triggered Immunity (ETI) that often –albeit not always (see below) culminate in Hypersensitive Response (HR), a rapid and localized cell death process thought to limit or preclude pathogens' growth [1], [2]. As a consequence of the gene-for-gene type of interaction linking these two components, plant R genes and their corresponding pathogen-encoded virulence factors evolve constantly and rapidly, so that HR, a common and ultimate manifestation of ETI, is usually only observed in specific plant species infected with specific pathogen strains. The plant hormones salicylic acid (SA), ethylene and jasmonic acid (JA) are crucially implicated in signaling networks underpinning both PTI and ETI [1], [2], [4], [5]; antimicrobial pathogenesis-Related Proteins (PRs), which include taumatine-like proteins and chitinases, are also often induced by both pathways and constitute, therefore, typical molecular markers of pathogen-induced defenses [6]. Although the occurrence of HR is classically used to discern PTI from ETI during bacterial or fungal infections [7], an HR-independent process known as Extreme Resistance (ER) is activated by a number of R proteins during ETI against viruses; ER is characterized by the lack of detectable accumulation of the triggering virus, and is accompanied by the onset of a broad-spectrum antiviral state in the absence of macroscopic or microscopic cell death lesions [8]–[11].

RETRACTED

RNA silencing is a conserved regulatory process that has evolved as an antiviral and antimicrobial defense mechanism in plants and animals [12]–[17]. Common features of RNA silencing across organisms include the involvement of double-stranded (ds)RNA as an initiator molecule, and accumulation of 21–24 nt small (s)RNAs that are processed from dsRNA by the RNAse III-like enzyme Dicer [18]–[20]. sRNAs are then incorporated into Argonaute (AGO)-containing effector complexes termed RNA-induced Silencing Complexes (RISCs) and, in case of extensive sequence complementarity between sRNA guide and target, AGO catalyses cleavage of the target RNA. *Arabidopsis thaliana* possesses four Dicer-like (DCLs) and ten AGO proteins [21], among which DCL4 and its surrogate DCL2, as well as AGO1 and AGO2, play essential roles as processors and effectors of virus-derived short interfering (si)RNAs, respectively [22]–[29]. DCL1- and AGO1-dependent micro (mi)RNAs produced from endogenous loci regulate the expression of many transcripts displaying miRNA sequence-complementarity, including mRNAs for transcription factors, enzymes, and regulators of PTI induced, notably, by bacteria [15]–[17], [30], [31].

As a consequence of these multiple RNA silencing-based defense layers, plant viruses, pathogenic bacteria, oomycetes and, possibly, fungi, have evolved suppressors of RNA silencing (SRs) that apparently target many steps of the siRNA and miRNA pathways [14], [32]–[37]. SRs are highly diverse in sequence, structure, and activity, and single SRs may target multiple points in RNA silencing pathways [14], [31]. Several viral SRs (VSRs) are known to affect AGO1 function [14]. For example, The *Beet western yellows virus* P0 protein was suggested to act as an F-box protein targeting AGO proteins for degradation, thereby preventing RISC assembly [38]–[40]. *Turnip crinckle virus* P38 was recently shown to bind directly and specifically AGO1 through mimicry of host-encoded glycine/tryptophane (GW)-containing proteins normally required for RISC assembly/function in diverse organisms [41], [42]. Physical sequestration of siRNAs is another common property of VSRs *in vitro* [43]–[47], although the extent to which this specific feature contributes to effective RNA silencing suppression *in vivo* remains unclear [42]. The most compelling example of active silencing suppression mediated by siRNA binding is provided by the tombusvirus P19 protein, of which the closely related *Tomato bushy stunt virus* (TBSV) and *Carnation Italian Ringspot virus* (CIRV; 97% identity) are the type representatives. Following its original discovery as a VSR [35], P19 was co-crystalized as a head-to-tail homodimer in direct association with an siRNA duplex [43], [48]. Supporting a direct and critical contribution of homodimerization and siRNA binding to the P19 VSR activity, stable point mutant alleles of the proteins lacking either property display complete loss-of-VSR-function phenotypes in both virus-infected and transgenic plants [43], [49]–[51]. sRNA binding by P19 also explains why its constitutive expression in Arabidopsis promotes developmental defects resembling those of plants carrying mutations in miRNA pathway components. Indeed, it was shown that P19 binds endogenous siRNAs and miRNAs, incurring, in the process, misregulation of the cognate endogenous targets of these molecules [42], [52].

RETRACTED

Remarkable parallels can be drawn between the general framework of silencing activation and its suppression by pathogens on the one hand, and the classical PTI-ETI scheme for resistance, on the other. This has prompted the suggestion that the two processes might be, in fact, manifestations of similar, if not identical, phenomena [31], [53]. In the case of (+)-stranded RNA viruses, for example, viral-derived dsRNA can be assimilated to a PAMP because this molecule is a mandatory product of viral replication. Similarly, the Dicer/AGO consortium orchestrating the antiviral reaction may be conceptually compared to the first defense layer underlying PTI [31]. Pursuing the comparison one step further and taking into account that VSRs are virulence effectors, it can be anticipated that the damages incurred by VSRs to the cellular silencing machinery may be sensed by host-encoded functions comprising, perhaps, dedicated R genes; the effects of such functions would thus be diagnosed, at least partly, by the typical outputs of ETI, including HR [31]. Supporting this notion, at least three VSR proteins from distinct virus families are known to trigger HR-like lesions in a host-specific manner [53]–[58]. It remains largely unknown, however, if these responses are stimulated by intrinsic silencing suppression properties or by other, unrelated functions of the viral proteins involved. Also unclear is whether virus resistance is effectively triggered upon recognition of these VSRs in these specific hosts, and to what extent the output of the induced defense compares with that of classical ETI.

RETRACTED

The present series of experiments was aimed at addressing these various issues using the well-characterized P19 VSR in tobacco. The results support the idea that RNA silencing and its suppression by viruses can be effectively rationalized within the frame of PTI-ETI, since we demonstrate, in authentic infection contexts, that (i) tombusviral virulence (ii) suppression of RNA silencing and (iii) induction of an ER-type of resistance with molecular features of ETI are all dependent upon the ability of P19 to bind sRNAs. Collectively, the data support the existence of host-encoded sensors that monitor the status/integrity of key RNA silencing components in plants. We propose, consequently, that perturbation of these components by pathogen-encoded SRs may activate potent ETI-like resistance responses. This proposed host counter-counter defensive layer likely constitutes an important driver in the evolution and diversification of SRs from viruses and perhaps other parasites.

## Results

### P19 is required to trigger an ETI-like resistance against TBSV in *N. tabacum*

TBSV P19 was shown to induce a HR-like response in *N. tabacum* and other *Nicotiana* species; a host-specific response strongly evocative of R gene-mediated ETI [54]–[57], To ascertain further if, indeed, P19 acts as an elicitor of immune responses, we generated transgenic *N. tabacum* cv. Xanthi lines expressing P19 under the GVG glucocorticoide inducible promoter, which is activated by dexamathazone (Dex::P19; [59]). The expression of P19 was quantified in two independent lines 0, 12 and 24 hours post Dex application (hpp); non-transgenic plants sprayed with DEX provided a negative control. While very low P19 transcript accumulation was observed before DEX treatment in the two transgenic lines, it was up to 4000 times higher following DEX application, at 12 and 24 hpp, compared to 0 hpp and to DEX-treated non-transgenic plants (Figure 1A). Accumulation of the P19 protein, mostly under homodimeric form, was also detected by Western analysis in the DEX-induced transgenic lines, but not in non-transgenic lines, using a polyclonal P19 antibody (Figure 1B). Accumulation of P19 following DEX induction correlated with the onset of three key markers of plant defense responses: (i) the progressive development of HR-like lesions in the sprayed areas of leaves, (ii) the accumulation of distinct PR proteins, PR1, PR2 and PR3, at 24 and 48 hpp (Figures 1C–D), and (iii) the accumulation of salicylic acid (SA) which was 4–5 times higher following DEX application at 24 hpp in the DEX-induced transgenic lines compared to 0 hpp and to DEX-treated non-transgenic plants (Figure S1). Collectively, therefore, the results presented in Figure 1 and Figure S1 suggest that in *N. tabacum*, P19 effectively acts as an elicitor of plant defense responses displaying at least superficial characteristics of ETI.

RETRACTED

**Figure 1:** DEX::P19 transgenic plants display defense responses following DEX application. (**A–B**) Leaves of five week old DEX::P19 transgenic and wild type plants (*N. tabacum* cv. Xanthi) were sprayed with DEX and the kinetics of P19 accumulation at transcript (A) and protein (B) levels was subsequently analyzed by qPCR and Western analysis, respectively. Actin was used as an internal control. (**C**) DEX::P19 transgenic or wild type plants were sprayed with DEX, and appearance of HR was assessed 5 days post-DEX application. We observed two and sometimes three bands for P19 dimers. These additional bands appear when P19 is expressed in *N. tabacum* but not in *N. benthamiana*. We believe that these additional bands are due to post-translational regulation of P19 by *N. tabacum*; this regulation might have a biological significance but evidence of this is not known yet. (**D**) PR protein accumulation at 0, 1 and 2 days post DEX application in wild type and DEX::P19 transgenic lines. Western analysis was conducted using anti-PR1, -PR2 and -PR3 antibodies. Coomassie or ponceau staining of the same extracts is shown to demonstrate equal protein loading. Experiments were repeated three times and showed similar results.

To test if P19 effectively induces resistance against TBSV in *N. tabacum*, Agrobacterium strains expressing either TBSV-GFP or TBSVΔP19-GFP, which is unable to express P19 [26], were used to inoculate leaves of 5-week old *N. tabacum*. At 5 days post-infiltration (dpi), virus accumulation was monitored under UV light via the appearance of green fluorescence in infiltrated leaves, and by Western analysis using an anti-GFP antibody. Viral replication was assessed directly in parallel by Northern analysis, using a GFP DNA fragment as a probe, which detects both genomic and sub-genomic RNAs of TBSV-GFP. We found that the presence or absence of P19 expression from TBSV-GFP had dramatically contrasted consequences on virus replication. Thus, GFP was not observed (Figure 2A–B) and the viral RNAs were below detection limits of Northern analyses (Figure 2C) in TBSV-GFP-inoculated leaves. In sharp contrast, however, both GFP accumulation and viral RNA replication were readily detectable in TBSVΔP19-GFP-infiltrated leaves at 5 dpi (Figures 2A–C). To further characterize the P19-mediated defense response, we used trypan blue staining as a diagnostic of cell death. Leaves were thus inoculated either with TBSV-GFP, P50 from *Tobacco mosaic virus* (TMV), which induces an HR in *N. tabacum* carrying the resistance gene N (as a positive control), or GUS as a negative control. We found that the visible and microscopic HR observed in P50-treated plants was absent from TBSV-GFP-infected and control leaves (Figure S2). These results strongly suggest that extreme resistance (ER) was triggered in TBSV-GFP-inoculated leaves of *N. tabacum*, and implicate, therefore, P19 as the elicitor of this defense. In fact, the results obtained here with P19 in tobacco are highly reminiscent of the well-studied interaction between *Potato virus X* coat protein (CP) and the Rx resistance protein in *Solanum tuberosum* or tobacco [8]. Indeed, while Rx typically confers ER to PVX in the context of authentic virus infections, isolated and prolonged production of CP, for instance *via* Agrobacterium-mediated transient expression, does trigger an HR in *Rx* potato genotypes [8], [9], as seen previously and here upon transient and transgenic expression of P19 in specific *Nicotiana* species (Figure 1B–C, [56]). With both PVX and TBSV, the potent antiviral state accompanying the ER (e.g. Figure 2C) probably stops virus replication before the CP or P19 have reached the levels required to trigger an HR [8], [9], a phenomenon presumably bypassed when both elicitors are produced in a virus replication-independent manner.

RETRACTED

**Figure 2:** P19 is required for extreme resistance of *N.* *tabacum* against TBSV. (**A**) Leaves of 5 weeks old *N. tabacum* cv. Xanthi plants were infiltrated with Agrobacterium expressing TBSV-GFP or TBSVΔP19-GFP. Pictures of infiltrated leaves were taken 5 dpi under transmitted light and UV. (**B**) GFP accumulation in infiltrated leaves from three independent plants. Western analysis was carried out using an anti-GFP antibody. Coomassie staining of the same extracts is shown to demonstrate equal protein loading. (**C**) Northern analysis of TBSV-GFP and TBSVΔP19-GFP RNA accumulation in infected plants at 5 dpi, using a GFP DNA fragment as a radioactive probe. Viral genomic and subgenomic RNAs are indicated; ribosomal RNA was used to demonstrate equal RNA loading. Experiments were repeated three times and showed similar results.

### Salicylic acid and ethylene are required for extreme resistance induced by P19

The potent (Figure 2C) and broad-spectrum [8] antiviral state triggered by ER is suspected to underlie the production of defense-related hormones, including SA, which possesses demonstrated antiviral activities [27], [60], [61]. The gaseous hormone ethylene is also important for induction of plant immunity [4]. To investigate the possible roles of these compounds in the ER-like resistance induced by P19 against TBSV, SA-deficient transgenic tobacco plants expressing NahG (Salicylate hydroxylase; [62]) and plants insensitive to Ethylene (ETR; [63]) were inoculated with TBSV-GFP using Agrobacterium-mediated delivery. At 5 dpi, leaves were observed under UV and samples were harvested for Western analysis using the anti-GFP antibody. Unlike WT plants, both transgenic plants failed to display resistance against TBSV (Figure 3A–B) and, accordingly, the P19-dependent induction of PR proteins was compromised in NahG plants ([64], [65]; Figure S3). Overall, these results indicate that SA and ethylene are required for the ER induced by P19 against TBSV. We then investigated if the HR-like lesions induced by P19 in tobacco leaves (Figure 1C) were SA- and/or ethylene-dependent. As seen in Figure 3C, necrosis was as extensive in leaves of NahG and ETR plants as it was in their non-transgenic counterparts at 5 dpi (Figure 3C), indicating that the HR triggered by P19, unlike the induced antiviral state, is neither SA- nor ethylene-dependent.

RETRACTED

**Figure 3:** Salicylic acid and ethylene are required for extreme resistance induced by P19 against TBSV. (**A**) Leaves of SA-deficient and ethylene-insensitive plants, or their corresponding WT counterparts, were infiltrated with *Agrobacterium tumefaciens* expressing TBSV-GFP. Leaves were observed under optical light and GFP fluorescence was visualized under UV at 5 dpi. (**B**) Western analysis was conducted to detect TBSV-GFP accumulation in the infiltrated leaves depicted in (A), using an anti-GFP antibody. Ponceau staining of the membrane is shown to demonstrate equal protein loading. (**C**) *A. tumefaciens* expressing P19 triggers an HR response is all depicted genotypes at 5 dpi. Experiments were repeated three times and showed similar results.

### sRNAs binding by P19 is necessary for P19-mediated elicitation of defense

Resolving the crystal structure of the P19-siRNA complex granted the identification of point mutations that debilitate the protein's VSR function without impacting its stability [43]. It was notably shown that a double mutation affecting tryptophan residues 39 and 42 (W39-42R) was sufficient to abolish siRNA binding by P19 *in vitro*, with the resulting stable mutant allele being unable to suppress RNA silencing *in planta* [43]. Using the same allele, we thus tested if the capacity of P19 to sequester siRNAs was required for the elicitation of ER in *N. tabacum*. We generated transgenic *N. tabacum* cv. Xanthi lines expressing CIRV P19W39-42R under the DEX inducible promoter (DEX::P19W39-42R). Expression of P19W39-42R was quantified in two independent lines 0, 12 and 24 hours after DEX application; transgenic line Dex::P19#1, expressing WT P19 (Figure 1B), was used as a reference for functional P19 levels in these experiments. Upon DEX application onto leaves of five week old plants, quantification of both mRNA (Figure 4A) and protein (Figure 4B) levels showed that accumulation of the P19 mRNA and of P19 homo-dimers was similar in the two independent DEX::P19W39-42R tobacco lines tested and in the Dex::P19#1 reference line (Figure 4A–B). Remarkably, P19W39-42R was neither able to induce SA accumulation, HR-like symptoms nor to promote accumulation of PR1, PR2 and PR3 compared to WT P19 (Figure 3C–D and Figure S1), suggesting that small RNA binding by P19 is necessary to trigger the onset of defense in *N. tabacum*. The results also show that defense elicitation can occur independently of virus infection, suggesting that binding of endogenous sRNAs by P19 is prerequisite for elicitation.

RETRACTED

**Figure 4:** Binding of small RNAs is mandatory for induction of plant immune responses by P19. (**A–B**) Leaves of five week old Dex::P19, Dex::P19W39-42R transgenic lines (*N. tabacum* cv. Xanthi) were sprayed with DEX and the kinetics of P19W39-42R accumulation at transcript (A) and protein (B) levels was analysed by qPCR and Western analysis, respectively. Actin was used as an internal control. (**C**) The transgenic lines described above were sprayed with DEX and appearance of an HR was assessed 5 day post-DEX application. (**D**) PR proteins accumulation at 0, 1 and 2 days post DEX application in Dex::P19 and Dex::P19W39-42R transgenic lines. Western analysis was conducted using anti-PR1, -PR2 and -PR3 antibodies. Coomassie or ponceau staining of the same extracts is shown to demonstrate equal protein loading. Experiments were repeated three times and showed similar results.

### RNA silencing suppression and sRNAs binding are not sufficient, *per se*, to trigger HR-like lesions in *N. tabacum*

The above results prompted us to investigate if silencing suppression via sRNA binding was sufficient, *per se*, to trigger the HR-associated defense response elicited by P19 in *N. tabacum*. To that aim, we used Agrobacterium strains producing various VSRs unrelated to P19. HcPro from *Tobacco etch virus*, P15 from *Peanut clump virus* and P21 from *Beet yellows virus* are all known to bind sRNAs *in vitro*, with high affinity for 21 nt-long species (Figure 5A; [45]). In the same *in vitro* assay, P14 from *Pothos latent virus* was shown to bind different sizes of sRNAs ranging from 21 nt to 26 nt, while P25 from PVX was, by contrast, devoid of sRNA binding activity (Figure 5A; [45]).

**Figure 5:** Effects of VSRs unrelated to P19. (**A**) List of VSRs used in this study alongside their preferential sRNA binding sizes, as established *in vitro*. P25 is unable to bind sRNAs *in vitro*. Leaves of five week-old *N. tabacum* cv. Xanthi were transiently infiltrated with *Agrobacterium tumefaciens* expressing either P19, P14, P15, P21, P25 or HcPro. (**B**) HR response as evaluated 5 days post infiltration of the various VSRs lsited in (A). (**C–D**) Leaves of *N. tabacum* cv. Xanthi were infiltrated with a mixture of Agrobacteria containing either P14, P15, P21 or HcPro together with a GFP transgene used as a visual and molecular reporter of the onset of RNA silencing in the co-infiltrated tissues. GFP fluorescence was visualized 4 days post-infiltration under UV light (C) and by Western analysis using an anti-GFP antibody (**D**). Ponceau staining of the same extracts is depicted to demonstrate equal protein loading. (**E**) Leaves of five week-old *N. tabacum* cv. Xanthi were infiltrated with *A. tumefaciens* strains expressing P19 in combination with either P14, P15, P21, HcPro, P25 or the GUS reporter gene. Appearance of P19-triggered HR lesions was monitored at 40 hpi (Left panel) and 96 hpi (Right panel). Experiments were repeated three times with similar results. (**F**) Western analysis of P19 protein levels in P19-VSR co-treatments. Proteins extracts from P19-VSRs or P19-GUS co-treated leaves were subjected to anti-P19 immunoblotting after 48 h. Ponceau staining of the membrane is shown to demonstrate equal protein loading. Experiments were repeated three times and showed similar results.

RETRACTED

We found that, unlike P19, neither of the above VSRs was able to trigger the HR-like response at 5 dpi following their transient expression in leaves of *N. tabacum* (Figure 5B). Nonetheless, in a well-established silencing suppression assay based on transient co-expression of a silencing GFP target transgene with VSRs [66], all of these proteins were clearly able to stabilize GFP accumulation, as assessed under UV illumination (Figure 5C) and by Western analysis (Figure 5D). By contrast, GFP accumulation remained low in tissues co-infiltrated with a control Agrobacterium strain expressing the GUS reporter gene (Figure 5C–D). Thus, all the VSRs tested were able to suppress GFP RNA silencing in this assay. The results indicate that the failure of the P19-unrelated VSRs to trigger an HR-like response cannot be explained by their inability to suppress RNA silencing in *N. tabacum*. Therefore, RNA silencing suppression is, in itself, insufficient to trigger this response. Moreover, given the documented high affinity of some of the VSRs used for siRNAs [42], [45], [67] the data suggest that sRNA binding *per se* is also insufficient to promote defense in *N. tabacum*. The most parsimonious interpretation of these results entails, therefore, that P19-mediated elicitation of host defenses in *Nicotiana* species involves the specific recognition of P19-sRNA complexes, or of downstream molecular events triggered by the specific association of both components.

RETRACTED

### Co-expression of unrelated VSRs compromise the onset of HR elicited by P19, but not resistance conferred by Rx against PVX

Even though none of the above-tested VSRs triggered, on its own, a defense response in *N. tabacum*, the intrinsic abilities of most of these proteins to bind sRNAs predicted that their co-expression with P19 would compromise the onset of HR-like lesions observed in Agrobacterium-infiltrated tissues (Figure 1C). As shown in Figure 5E, this was indeed the case: the appearance of necrotic tissues was significantly delayed and less extensive at 96 hours in leaf patches that had received the P19-VSR co-treatments compared to leaves co-treated with P19 and GUS as a negative control (Figure 5E). Remarkably, the delayed onset of HR was not observed in co-treatments involving P19 and the P25 protein of PVX, which, unlike all the other VSRs tested, does not bind sRNAs *in vitro* ([45]; Figure 5E). Western analyses employing a P19 antibody also confirmed that the delayed onset of HR was unlikely to be a consequence of altered levels of P19 homodimers in the P19-VSR co-treated leaves, compared to control leaves (Figure 5F).

Given that P14, P15, P21 and Hc-Pro are all known to bind sRNA, at least *in vitro* [45], we assessed whether the compromised HR-like cell death phenotype observed upon concomitant expression of P19 with these VSRs resulted from a direct competition for sRNA binding, potentially decreasing the amount of P19-siRNA complexes. To address this point we transiently expressed, in *N. benthamiana*, a HA-tagged version of P19 (P19HA), either alone or in combination with P15 or P21 (Figure 6). As a source of siRNAs, we used a 35S promoter-driven inverted-repeat (IR) construct, corresponding to the 5′ part (‘GF’) of the GFP sequence, which is processed into 21 nt- and 24 nt-long siRNAs. Northern analysis of the sRNA fraction of P19HA immunoprecipitates showed that, as expected, P19 specifically bound the 21 nt-long GF siRNAs. Both P15HA and P21HA displayed the same 21 nt siRNA size preference as P19 for binding. However, P21 sequestered 21 nt siRNAs significantly more efficiently than the two other VSRs, as shown by the much stronger signal detected in P21HA immunoprecipitates (Figure 6). This most likely explains the decreased GF siRNA levels observed in P19HA and P15HA immunoprecipitated fractions when these VSRs were concomitantly expressed with P21 (Figure 6). However, in contrast to P21, P15 did not alter the amount of siRNA bound by P19 whereas P19 prevented P15 siRNA binding and competed with P21 siRNA binding (Figure 6). Therefore, in the case of P15, the compromised P19-triggered HR-like cell death phenotype is unlileky to result from a reduction in the amount of formed P19-siRNA complexes. Overall, these results show that, although necessary, the sRNA binding capacity of P19 is not sufficient for host defense elicitation in *N. tabacum*, suggesting that the onset of ER is intrinsically linked to the VSR function of P19 and not just the formation of P19-siRNA complexes *per se* (Figure 3).

RETRACTED

**Figure 6:** Differential effects of co-expressed VSRs on P19 siRNA-binding capacity. (**A**) RNA gel blot analysis of GF siRNA accumulation (@GF) in total RNA and HA immunoprecipitated fractions from *Nicotiana benthamiana* infiltrated leaves expressing HA-tagged P15, P19 or P21 VSRs, either alone (-) or in combination with untagged VSRs. Ethidium bromide staining of ribosomal RNA (rRNA) is used as loading control. (**B**) Protein blot analysis of HA-tagged VSRs accumulation (@HA) in total (input) or immunoprecipitated fractions (IP@HA) of the samples described in (A). Coomassie staining of the membrane was used to verify equal loading after western blotting. EV: empty vector. Experiments were repeated three times and gave similar results.

To further ascertain this idea, we took advantage of the fact that Rx-mediated ER is triggered by the PVX-encoded CP protein, which does not display any intrinsic VSR activity [68]. Moreover, Rx-mediated ER can be recapitulated in transgenic *N. tabacum* upon inoculation of PVX-GFP using leaf-infiltration of Agrobacterium. We reasoned that, unlike in the above example where resistance was highly dependent upon the VSR function of the P19 elicitor, Rx-mediated resistance would remain unaffected by co-expression of VSRs with PVX-GFP. As shown in Figure 7, accumulation of Agrobacterium-delivered PVX-GFP was abolished in leaves of plants expressing transgenic Rx, compared to non-transgenic plants. Furthermore, this pattern remained unaffected by transient co-expression of HcPro, P21, P15 P14 VSRs, or a control GUS transgene (Figure 7).

**Figure 7:** VSRs that bind small RNAs *in vitro* do not compromise resistance mediated by Rx against PVX. Leaves of five week-old *N. tabacum* expressing the Rx gene and its corresponding counterpart lacking this R gene was infiltrated with of *A. tumefaciens* strains expressing PVX-GFP together with a strain expressing P14, P15, P21, P25, HcPro or the GUS reporter gene. GFP accumulation in infiltrated leaves was detected by Western analysis using an anti-GFP antibody. Ponceau staining of the membrane is shown to demonstrate equal protein loading. Experiments were repeated three times and gave similar results.

RETRACTED

## Discussion

Cross-talk between RNA silencing pathways and both PTI and ETI pathways has been established experimentally in the case of bacterial pathogens [12], [15]. In all cases so far, PAMP recognition activates endogenous RNA silencing pathways to target negative regulators of disease resistance, leading to potentiation of basal defense [12], [15], [31]. Bacterial-encoded SRs, in turn, target this basal defense by inhibiting various, and perhaps multiple, steps of host silencing pathways.

The work presented here describes how the activity of the viral suppressor P19 is sensed in specific *Nicotiana* species to induce immunity against the P19-producing virus. This immunity displays several key attributes of ETI, including the involvement of SA and ethylene, as well as the production of PR proteins. The timing of P19 homodimers accumulation correlates with the extent of cell death and PR proteins production; this is in agreement with data showed previously in which the authors used the same inducible promoter as the one we used in this study [69]. Remarkably, antiviral immunity is also accompanied by a lack of visible HR-like lesions, at least in the context of authentic tombusvirus infection, a phenomenon highly reminiscent of extreme resistance (ER) observed, for instance, during the CP-Rx interaction in PVX-infected plants. Further supporting the analogy between P19-mediated defense and the ER triggered by Rx, strong and isolated expression of their respective elicitors (i.e. P19 or CP, respectively) promotes the appearance of HR-like lesions in both cases. Nonetheless, a marked difference between the Rx-CP and the P19 systems is the reliance of the latter upon RNA silencing suppression, a function not associated with the CP of PVX [68].

Our findings were, in fact, not completely unprecedented. Hence, the P38 capsid protein of *Turnip crinkle virus* binds AGO to inhibit its loading with sRNAs [41], [42], [70]. P38 was also shown to induce HR-associated defense responses in the Arabidopsis ecotype Dijon-0 and its inbred derivative Dijon-17 [71], [72], a level of host specificity that strongly evokes an ETI-type of response. The elicitor of the *N* resistance gene, which confers ETI to TMV, had been also mapped to the p50 helicase subunit of the viral replicase, p126. Remarkably, the same domain of p126 was recently identified as being sufficient to suppress RNA silencing in *N. benthamiana* [73]. Moreover, the helicase enzymatic activity of p50 was found dispensable for both N-mediated resistance and silencing suppression, suggesting that the VSR activity of P50 might stimulate ETI via the activation of N. Seminal work carried out more than a decade ago also provided key insights into the potential contribution of the 2b protein from *Tomato aspermy cucumovirus* (TAV2b) to the induction of ETI, possibly through its VSR activity. Indeed, when expressed from recombinant TMV, TAV2b was found to activate strong host resistance in tobacco, typical of the gene-for-gene interaction linking R proteins to their elicitors [53]. Moreover, the N-terminal region of TAV2b was found critical for both VSR activity and resistance elicitation, suggesting that the same or overlapping domains of the protein are involved [53]. Interestingly, Chen et al. [74] recently showed that Tav2b effectively binds sRNAs, highly reminiscent of the situation presented here with P19.

RETRACTED

The seminal observation made with TAV2b led the authors to suspect that RNA silencing and its suppression on the one hand, and ETI on the other, were probably linked phenomena, at least in some cases; this view became strongly substantiated through subsequent work conducted with plant pathogenic bacteria (reviewed in [31]). The data obtained in this manuscript add further strength to this idea by showing the importance of RNA silencing suppression in the resistance mediated by P19, because immunity to TBSV was only achieved if the protein retained its capacity to suppress gene silencing, for which sRNA binding is a prerequisite. We suspect that the reported ETI-like response triggered by P19 in the absence of visible HR might also strongly contribute to its additional, albeit poorly understood, role as a host-specific determinant of systemic viral movement [51], [75]. This hypothesis is particularly appealing given the involvement of SA and ethylene in the P19-elicited response in *N. tabacum*. Indeed both hormones are known to mediate, directly or indirectly, systemic, in addition to localized, defense responses.

Immune signaling pathways seem to be widely conserved across fungal, bacterial and viral interactions that lead to ETI in plants. The fact that P19-mediated resistance was compromised by many unrelated VSRs, unlike resistance activated by Rx argues, therefore, against an interference at the level of disease resistance signaling. Moreover, the PVX coat protein (elicitor of Rx) does not possess VSR function [68]. The fact that the integrity of the P19 binding domain is required for defense elicitation, together with the failure of PVX P25, among the VSR tested here, to alter the P19-mediated HR response, suggests that sRNA binding, required for VSR function, is a key component for defense activation in *N. tabacum*. It is, however unlikely to be sufficient, because none of the other VSRs tested was able to recapitulate, on its own, the defense phenotype induced by P19 when transiently expressed, despite that many of them bind sRNA *in vitro* and probably *in vivo*. Additionally, P15 could suppress the P19-mediated HR even though it did not outcompete P19 for siRNA binding in the *N. benthamianan* transient expression assay. The simplest interpretation of these results, therefore, is that P19 dimers complexed with sRNAs initiate a signal that is specifically sensed in *N. tabacum* to trigger extreme resistance against TBSV or that a conserved motif or structure important for sRNA binding by P19 is sensed in the plant. A non-mutually exclusive possibility holds that sensing occurs downstream, as a consequence of specific P19-sRNA association in a manner suppressed by the action of VSRs such as P15, which may share downstream silencing targets with P19 including AGOs. Interestingly, HR-like lesions and *PR* proteins accumulation could be triggered by P19 in the absence of a viral infection, suggesting that endogenous sRNAs, including siRNAs and miRNAs, which are effectively bound by P19 together with viral-derived siRNAs during infection [43], [49], [67], [76], form one component of the trigger. Hence, a recent study in transgenic Arabidopsis shows that binding of endogenous miRNAs by VSRs is much less widespread than was originally anticipated. In fact, P19 was, among many VSRs tested (including several used in the present study), the only protein to prevent loading of miRNAs into AGO1. By contrast, all of the VSRs tested could effectively prevent loading of exogenous siRNAs into AGO1 [42]. This peculiarity may contribute to explain the specific ability of P19 to trigger HR-like lesions and ER in *N. tabacum*. It is also possible that the binding of P19 to si/miRNAs promotes a specific change in the integrity or conformation of silencing effector proteins, including AGOs, and that these changes are sensed in a host-specific manner.

miRNAs have roles in plant basal and race-specific resistance against bacterial pathogens [15], [16], [77]. Furthermore, some plant miRNAs appear to have evolved to control R gene expression presumably to prevent the known fitness cost of their constitutive expression in the absence of pathogens [78]–[80]. For example, nta-miR6019 (22-nt) and nta-miR6020 (21-nt) guide the cleavage of the TIR-NB-LRR *N* transcript from tobacco, which confers resistance to *Tobacco mosaic virus* [79]. Likewise, Sl-miR482 attenuates expression of a large family of NBS-LRR genes from tomato and its accumulation is decreased in plants infected with *Turnip crinkle virus*, *Cucumber mosaic virus*, *Tobacco rattle virus* and *Pst* DC3000 [80]. Therefore, given the above context, miRNA sequestration by P19 might generally enhance host immune responses induced by virulent and avirulent pathogens. Interestingly, however, miR168, which targets the antiviral silencing effector AGO1, is specifically not sequestered and, in fact, induced by P19, suggesting that, in this case, miRNA binding by P19 favours viral infection without activating immune responses [81].

RETRACTED

We have shown here, with the P19-*N. tabacum* model, that the general scheme of silencing induction and suppression by plant viruses can be readily accommodated within the classical frame of ETI/PTI. In particular, our study sheds light on an additional layer of defense, whereby hosts can sense and respond to the damages caused by VSRs to the cellular silencing machinery. The existence of this additional layer is also consistent with the fast evolving and highly diverse nature of VSRs. Indeed, potent host counter-counter-defense measures probably impose strong selective pressure on pathogens to accelerate or refine the modeling of their virulence factors, thereby contributing further to the never-ending arms race opposing parasites to their hosts. A future challenge will be to assess the extent to which the phenomenon described here is shared not only among plant-virus, but also plant-bacteria, plant-fungal and plant-oomycetes interactions, and how elucidation of its biochemical and genetic underpinnings might improve our understanding of PTI and ETI at large. Finally, and most importantly, a strong -albeit still speculative- implication of our results is the existence of dedicated host-encoded R proteins that should monitor the status of key RNA silencing components in plants, and perhaps other organisms. Identifying these elusive silencing-associated R proteins and their guardees would certainly constitute a major breakthrough in the field.

## Materials and Methods

### Plant conditions and transgenic lines

Wild type and transgenic plants were grown under conditions of 8 h darkness at 19°C, 16 h light at 22°C, with 70% relative humidity. Independent tobacco (*N. tabacum*) transgenic lines carrying the wild type P19 and its mutant P19W39-42R under Dex inducible promoter [59] were generated using the *Agrobacterium tumefaciens* leaf disc transformation method [82]. The disarmed pTA7001-Dex-P19, pTA7001-Dex-P19W39-42R were used for transformation. The transgenic plants generated were named Dex::P19 and Dex::P19W39-42R.

RETRACTED

### Transient expression

*A. tumefaciens* strains containing the constructs P19 [35], P25 [68], P15 [83], HcPro [67], P14 and P21 [45] were grown overnight at 28°C in Lauria Bertani (LB) broth supplemented with 50 µg/ml kanamycine, 10 µg/ml rifampicine and 25 µg/ml gentamycine. Bacterial cultures were then pelleted at 4 500× *g* for 15 min and the supernatant was discarded. Pellets were resuspended in 10 mM MgCl_2_ supplemented with 200 µM acetosyringone and brought to an OD 0.5. These bacterial suspensions were infiltrated in the plant leaves using a syringe. Co-agroinfiltration of mGFP and VSRs were done at 0.5 OD.

### Protein extraction and gel blot analysis

For transgenic plants, a solution of 25 µg/ml Dexametasone supplemented with 0.1% v/v Silwet L-77 was sprayed onto leaves of 5 week-old transgenic plants. Samples were harvested at 0, 12, 24 and 48 hours after DEX application, immediately frozen in liquid nitrogen, and kept at −80°C before extraction.

Total proteins were extracted from 100 to 200 mg of homogeny of frozen leave 200 µl of extraction buffer [25 mM Tris-HCl pH 7.5, 1 mM EDTA, 150 mM NaCl, 10% glycérol, 5 mM dithiothreitol (DTT)] and a protease inhibitor cocktail (Sigma). The crude extract was centrifuged at 12000 g for 15 min. The supernatant was kept and total proteins were quantified by Bradford assay (Bio-Rad Laboratories, Ontario). Samples were diluted in Leammli buffer and boiled for 5 minutes before separation on 12% SDS-PAGE. 50 µg of proteins of each sample was used for Western analysis. Proteins were subjected to gel blot analysis using a rabbit polyclonal PR1, PR2 or PR3 antibodies, at a dilution of 1 : 8000 [84]. For detection of the GFP, a rabbit polyclonal IgG antibody was used at 1/3000 (GFP (FL), sc-8334, Santa Cruz Biotechnology). For detection of P19, we used an affinity purified rabbit polyclonal IgG antibody obtain from GeneScript and raised against a synthetic peptide of the P19 protein (GNDAREQANSERWDC). It was used at 1/300. Coomassie Blue or red ponceau staining were used to confirm equal protein loading. Horse Radish Peroxidase-conjugated anti-rabbit IgG was used as secondary antibody at 1 : 14500 (Sigma Aldrich). Immunodetection was conducted with chemiluminescent substrate (Bio-Rad, immun-star kit) followed by X-ray film exposure.

### Quantitative PCR

Total RNA was extracted from tobacco tissues using the RNeasy Plant Mini Kit (Qiagen Science, Maryland, USA) according to the manufacturer's instructions. 2 µg of each RNA samples were reverse transcribed into cDNA using SuperScript II reverse transcriptase (Invitrogen). Samples were diluted 1/5 in DEPC water and qPCR was performed using POWER SYBR Green (Applied Biosystems, Warrington, UK) according to the manufacturer's instruction. Primers used were: qPCR NTAC1F 5′-CTGTACTACTCACTGAAGCACCTC-3, qPCR NTAC1R 5′- GGCGACATATCATAGCAGGA -3, qPCR P19F 5′-TTGGTTTCAAGGAAAGCTG-3, qPCR P19R 5′-GATCCAAGGACTCTGTGCA-3, qPCR1.

RETRACTED

### Virus infections

*A. tumefaciens* strains containing the constructs 35S::TBSV-GFP or 35S::TBSVΔP19-GFP (Kindly provided by Herman B. Scholthof [26]) were grown overnight at 28°C in Lauria Bertani (LB) broth supplemented with 50 µg/ml kanamycine, 10 µg/ml rifampicine and 25 µg/ml gentamincin. Bacterial cultures were then pelleted at 4 500× *g* for 15 min and the supernatant was discarded. Pellets were resuspended in 10 mM MgCl_2_ brought to 0.5 OD and supplemented with 200 µM acetosyringone. Bacterial suspensions were then incubated at room temperature for 1–3 hours before being infiltrated into young leaves of 5 week-old *Nicotiana tabacum* plants, using a syringe. Inoculated plants were grown under conditions of 8 h darkness at 18°C, 16 h light at 20°C with 70% relative humidity. Viral infection was monitored over time under U.V. illumination and samples were collected at 6 dpi, frozen in liquid nitrogen and kept at −80°C before extraction of protein or RNA. *A. tumefaciens* strain containing the construct 35S::PVX-GFP [85] was used for PVX assays. Infections were conducted as described above, except that the final OD used was 0.25. VSR were co-agroinfiltrated at final OD of 0.25.

### Northern analysis

Total RNA was extracted using TRI reagent (Sigma), precipitated with isopropanol and the RNA pellet was resuspended in 50% deionized Formamide. Analysis was performed as described [66]. The signal was detected using X-ray films.

### Trypan blue staining

Sample were boiled for 5 minutes in the staining solution [10 ml of lactic acid, 10 g of phenol, 10 ml of glycerol, 10 ml of water, 10 mg of trypan blue, mixed 1∶1 with ethanol]. Samples were then destained using chloral hydrate as previously described [86], [87].

### Immunoprecipitation experiments

The cassettes for transient expression of GFFG dsRNA and silencing suppressors have been described previously [66], [67]. Agrobacterium-mediated transient expression in *N. benthamiana* leaves was as described previously [88].

For immunoprecipitation experiments, 400 mg of frozen tissue harvested 5 days post-infiltration was ground in liquid nitrogen and homogenized in 3 ml/g of extraction buffer (50 mM Tris–HCl, pH 7.5, 150 mM NaCl, 10% glycerol, 0.1% NP-40 and complete protease inhibitor cocktail (Roche) for 30 min at 4°C. Cell debris was removed by centrifugation at 12000 g at 4°C for 30 min. Extracts were pre-cleared by incubation with Protein A-agarose (Roche) at 4°C for 1 h. Pre-cleared extracts were then incubated with anti-HA polyclonal antibody (Sigma) and protein A-agarose overnight at 4°C. Immunoprecipitates were washed three times (15 min each) in extraction buffer. Aliquots of the inputs and immunoprecipitates were collected for protein blot analysis. For RNA analysis, immune complex were subjected to Tri-Reagent extraction (Sigma).

RETRACTED

### Salicylic acid quantification

An amount of one to one v/w of cold 80% MeOH was added to finely ground plant tissue (300–500 mg) for extraction of phenolic compounds. Samples were vortexed then shaken overnight at 4°C. The following morning, the samples were vortexed and centrifuged 16,000 g for 10 min. The supernatant was transferred to a new Eppendorf tube, filtered through a 0.22-µm syringe filter and 50 to 100 µl injected into HPLC. Samples were injected using Waters 2695 separation module (Waters Corp.) and a Lichrospher RP-18 (5 µm) column (4 mm×250 mm) at 30°C, and compounds detected with a Waters 996 diode array scanning 200 nm–400 nm, followed, in tandem, by a Waters 2475 Fluorescence detector, with an excitation wavelength of 290 nm emission and a scan of 300–500 nm. The maximum expected emission for free salicylic acid using this excitation wavelength was at 390–400 nm. The HPLC system was controlled and data analysed with the Empower2 software. Standard free salicylic acid (Sigma 84210) standards were prepared at 100 ng/ml, 250 ng/ml, 500 ng/ml, 1000 ng/ml and injected under the same conditions. The solvents were acidified water (solvent A: 0.1% Phosphoric acid in nanopure water) and acetonitrile HPLC grade (solvent B) with an elution flow rate of 1 mL/min. The gradient used was as follows: time (min)/%A/%B: 0/100/0, 5/95/5, 10/95/5, 14/90/10, 20/80/20, 23/80/20, 30/65/35, 35/65/35, 43/50/50, 48/25/75, 55/0/100 and 60/0/100. The injected volume was 50 µL for each sample. Three biological replicates for each treatment/time point were extracted and injected independently into the HPLC. Linear regressions were generated between compound concentration (independent variable) and peak areas (dependent variable). The equations obtained were used to calculate the concentration of each phenolic compound in the analyzed samples. Every sample was also spiked with 0.8 µg/ml free salicylic acid and injected independently to confirm the quantities determined by the software.

## Supporting Information

Figure S1 **P19-mediated accumulation of SA in** ***N. tabacum*** **requires its capacity to bind sRNAs.** Five-week-old WT, Dex::P19 and Dex::P19W39-42 plants were sprayed with Dex and samples were harvested at 0 and 24 hours post treatment (hpt) for SA quantification. Error bars represent the SD (n = 3). Experiments were repeated two times and gave similar results.
(TIF)

Figure S2 **TBSV does not induce microscopic HR in** ***N. tabacum*** **.** (A–B) Five week-old *N. tabacum* cv. Xanthi plants were transiently infiltrated with a solution of *A. tumefaciens* expressing either GUS, TBSV-GFP or P50 and 3 and 5 dpi leaves were stained with trypan blue to see macroscopic (A) and microscopic HR using an Zeiss Axioskop microscope (Zeiss AxioCam MRc with the Axiovision Rel. 4.8 program) under bright-field illumination (B). Experiments were repeated at least three times and gave similar results.
(TIF)

Figure S3 **P19-mediated, SA-dependent immune responses are compromised in NahG plants.** Leaves of five weeks old tobacco wild type and NahG plants were transiently infiltrated with a solution of *A. tumefaciens* expressing P19 (0.25 OD in MgCl_2_ 10 mM). The accumulation of acidic PR3 and PR5 proteins was monitored by western blot 3 days post agroinfiltration of both, wild type and *nahG* plants. Lower panel shows Ponceau Red staining of ribulose-1,5-biphosphate carboxylase/oxygenase (Rubisco) for confirmation of equal loading. Experiments were repeated three times and showed similar results.
(TIF)
